The article "Influence of Early Predictive Nursing on Complications and Quality of Life in Patients after Colorectal Cancer Surgery" was retracted in 2023. Reasons: unreliable results or conclusions; lack of ethics approval or compliance; concerns about the data; concerns about the peer review.

# Influence of Early Predictive Nursing on Complications and Quality of Life in Patients after Colorectal Cancer Surgery

**DOI:** 10.1155/2022/8410664

**Published:** 2022-06-08

**Authors:** Jing Gao, Qiuyang Zhang, Xiaolin Zhao, Wei Gao

**Affiliations:** ^1^Nursing Support Center Department, First Affiliated Hospital of Harbin Medical University, Harbin, Heilongjiang, China; ^2^Nursing Department, First Affiliated Hospital of Harbin Medical University, Harbin, Heilongjiang, China; ^3^Nucleic Acid Collection Room, First Affiliated Hospital of Harbin Medical University, Harbin, Heilongjiang, China; ^4^Outpatient Center Operating Room, First Affiliated Hospital of Harbin Medical University, Harbin, Heilongjiang, China

## Abstract

**Objective:**

To analyze the effect of early predictive nursing on complications and quality of life in patients after colorectal cancer surgery.

**Methods:**

A total of 130 patients with colorectal cancer who were diagnosed and underwent surgical resection in our hospital from 2019 to 2021 were recruited and assigned via the random number table method (1 : 1) to receive either conventional nursing (routine group) or predictive nursing (study group). Outcome measures included the incidence of complications and the quality of life.

**Results:**

Predictive nursing was associated with shorter operation time and hospital stay and less blood loss (2.35 ± 0.41, 9.32 ± 1.86, and 70.52 ± 16.52) versus conventional nursing (3.02 ± 0.78, 11.20 ± 2.14, and 81.51 ± 17.74) (all *P* < 0.05). Patients in the study group showed a lower incidence of complications than the control group (10.76% vs 35.38%) (all *P* < 0.05). Predictive nursing resulted in better anxiety relief than conventional nursing (*P* < 0.05). Predictive nursing was associated with higher emotional function, cognitive function, role function, and physical function scores (83.51 ± 12.56, 82.45 ± 9.15, 82.48 ± 10.46, 84.43 ± 13.48, and 82.73 ± 9.67) than conventional nursing (73.85 ± 13.54, 72.54 ± 12.74, 72.48 ± 10.45, 73.99 ± 14.51, and 72.45 ± 11.69) (all *P* < 0.05). Patients receiving predictive nursing showed a significantly higher nursing satisfaction versus conventional nursing (*P* < 0.05).

**Conclusion:**

Early predictive nursing for patients receiving colorectal cancer surgery can lower the incidence of complications, effectively improve the quality of life of patients, shorten the hospital stay, reduce the amount of bleeding, and enhance the satisfaction of patients.

## 1. Introduction

Colorectal cancer (large intestine cancer) [1] is a common malignant tumor of the digestive tract. Statistics show that colorectal cancer is the third most common malignant tumor in the world and the second most common cause of death from malignant tumors [2, 3]. According to the GLOBOCAN project of the WHO *Cancer* Research Center [4], the number of new cases of colorectal cancer worldwide in 2018 is about 1.8 million, and the number of deaths is about 880,000. Previous research has shown that the onset of colorectal cancer is related to factors such as age, region, and gender [5]. Most of the clinical symptoms in the early stage are atypical symptoms such as indigestion and fecal occult blood, which usually results in the development of the disease to an advanced stage by the time of diagnosis [6, 7]. Clinically, the key to the diagnosis and treatment of colorectal cancer is early diagnosis and treatment, and surgery is the main treatment method [8]. Radical resection is effective for patients in the early stage of cancer, while those in the advanced stage require postoperative adjuvant chemotherapy and radiotherapy [9] to obtain a better therapeutic effect. However, the invasiveness of surgery results in trauma and a certain risk of postoperative complications, which may compromise the prognosis [10, 11].

Currently, the efficiency of conventional postoperative nursing is considered unsatisfactory for patients [12], so high-quality nursing is a key factor to improve nursing satisfaction. High-quality nursing for patients undergoing surgery is an inevitable development of routine nursing interventions for the advancement of the healthcare system [13]. Predictive nursing is a new type of nursing method and refers to the comprehensive analysis of the patient's condition, the identification of potential risks in advance, and the application of effective nursing measures to prevent nursing risks and improve the nursing efficiency [14]. Accordingly, this study aims to analyze the impact of early predictive nursing on the complications and quality of life of patients undergoing colorectal cancer surgery to provide a clinical reference.

## 2. Materials and Methods

### 2.1. Baseline Data

A total of 130 patients with colorectal cancer who were diagnosed and underwent surgical resection in our hospital from 2019 to 2021 were recruited and assigned via the random number table method (1 : 1) to receive either conventional nursing (routine group) or predictive nursing (study group). In the routine group, there were 37 males and 28 females, aged 42–73 years, with a disease duration of 1–4 years. In the study group, there were 36 males and 29 females, aged 41–75 years, with a disease duration of 1–4 years.

### 2.2. Inclusion and Exclusion Criteria

Inclusion criteria are as follows: (1) all patients were diagnosed with rectal cancer by pathological examination; (2) with normal coagulation function; (3) with complete clinical data.

Exclusion criteria are as follows: (1) with severe liver and kidney insufficiency; (2) with severe multifunctional organ failure or arrhythmia; (3) with allergies to the drug used in the present study.

### 2.3. Nursing Methods

Patients in the routine group received routine care, including preoperative examination, health education, postoperative care, physical sign monitoring, and discharge health guidance [15].

The patients in the study group were given predictive nursing. (1) Psychological intervention: the patients were given psychological counseling for treatment to eliminate their negative emotions, enhance their confidence in treatment, and improve their treatment compliance. (2) Dietary care: before surgery, a reasonable dietary plan was formulated for the patients according to their individual differences. The patients fasted for 3–5 days after surgery, and liquid food was allowed after exhaustion. Their intake and output were recorded and their condition was monitored to maintain water and electrolyte balance. Normal diet can be gradually restored, vitamins and high protein were timely and sufficiently supplemented, and overeating was prevented. (3) Intraoperative intervention: the patients' intraoperative physical signs were strictly monitored. After the signs were stable, the supine position was changed to a semirecumbent position to relieve the patients' discomfort. Other interventions included gastrointestinal decompression, drainage fluid monitoring, and complication prevention care to facilitate postoperative recovery. (5) Follow-up: after discharge from the hospital, all patients were followed up regularly, and the postoperative recovery status of the patient was timely recorded. The patients were instructed to perform proper exercises according to their physical tolerance, such as walking, gymnastics, and Taichi. The patients were also provided with medication and dietary guidance.

### 2.4. Evaluation Criteria

(1) The operation time, blood loss, and hospitalization time of the two groups of patients were recorded and compared.

(2) The occurrence of complications in the two groups was recorded, including abdominal distension, hypothermia, incision infection, subcutaneous emphysema, and lower extremity venous thrombosis. The total incidence of complications in the two groups was calculated and compared.

(3) The negative emotions of the two groups of patients were evaluated by the Self-rating Anxiety Scale (SAS) [15]. The total score on the SAS scale was 100 points. A score of 50–70 points indicates mild anxiety, a score of 71–90 points indicates moderate anxiety, and a score over 90 points indicates severe anxiety.

(4) The EORTC Quality of Life Questionnaire-Core 30 (EORTCQLQ-C30) [16] was used to evaluate the quality of life of the two groups of patients before and after treatment, including 30 items, 5 functional areas (social function, emotional function, cognitive function, role function, physical function). The higher the score, the better the patient's quality of life.

(5) Nursing Satisfaction Questionnaire created by our hospital was used to assess the patients' nursing satisfaction, which was divided into four levels (highly satisfied, satisfied, less satisfied, and dissatisfied).

### 2.5. Statistical Analysis

GraphPad Prism 8 software was used for image rendering, and SPSS 22.0 software was used for data analyses. Count data (n (%)) and measurement data (*X* ± *s*) were subjected to chi-square and *t*-tests, respectively. The rank sum test was used for comparison of the grade data. Differences were considered statistically significant at *P* < 0.05.

## 3. Results

### 3.1. Baseline Data

There was no significant difference in general data between the two groups of patients (see Table 1).

### 3.2. Surgical Indices

Predictive nursing was associated with shorter operation time and hospital stay and less blood loss (2.35 ± 0.41, 9.32 ± 1.86, and 70.52 ± 16.52) versus conventional nursing (3.02 ± 0.78, 11.20 ± 2.14, and 81.51 ± 17.74) (all *P* < 0.05, Table 2).

### 3.3. Complications

In the routine group, there were 5 (7.69%) cases of abdominal distension, 5 (7.69%) cases of hypothermia, 4 (6.15%) cases of incision infection, 6 (9.23%) cases of subcutaneous emphysema, and 3 (4.62%) cases of lower extremity venous thrombosis. In the study group, there were 3 (4.62%) cases of abdominal distension, 1 (1.54%) case of hypothermia, 1 (1.54%) case of incision infection, 2 (3.08%) cases of subcutaneous emphysema, and 0 (0.00%) case of lower extremity venous thrombosis. Patients in the study group showed a lower incidence of complications versus the control group (10.76% vs 35.38%) (all *P* < 0.05) (see Table 3).

### 3.4. Negative Emotions

In the routine group, there were 29 (44.61%) cases of normal psychological status, 23 (35.38%) cases of mild anxiety, 8 (12.31%) cases of moderate anxiety, and 5 (7.69%) cases of severe anxiety. In the study group, there were 48 (73.84) cases of normal psychological status, 16 (24.62%) cases of mild anxiety, 1 (1.54%) case of moderate anxiety, and 0 (0.00%) cases of severe anxiety. Predictive nursing resulted in better anxiety relief versus conventional nursing (*Z* = 1.475, *P* < 0.05).

### 3.5. Quality of Life Score

Before the intervention, there was no significant difference in the scores in various areas of the quality of life between the two groups (*P* < 0.05). Predictive nursing was associated with higher emotional function, cognitive function, role function, physical function scores (83.51 ± 12.56, 82.45 ± 9.15, 82.48 ± 10.46, 84.43 ± 13.48, and 82.73 ± 9.67) than conventional nursing (73.85 ± 13.54, 72.54 ± 12.74, 72.48 ± 10.45, 73.99 ± 14.51, and 72.45 ± 11.69) (all *P* < 0.05) (see Table 4).

### 3.6. Patient Satisfaction

In the routine group, 17 (26.15%) cases were highly satisfied, 23 (35.38%) cases were satisfied, 19 (29.23%) cases were less satisfied, and 6 (9.23%) cases were dissatisfied, with an overall satisfaction rate of 40 (61.54%). In the study group, 30 (46.15%) cases were highly satisfied, 32 (49.23%) cases were satisfied, 3 (4.61%) cases were less satisfied, and 0 (0.00%) was dissatisfied, with an overall satisfaction rate of 62 (95.38%). Patients receiving predictive nursing showed a significantly higher nursing satisfaction versus conventional nursing (*P* < 0.05) (see Figure 1).

## 4. Discussion

Colorectal cancer is the third most common malignant tumor worldwide and the second most common cause of death from malignant tumors. Previous studies have shown an increasing incidence of colorectal cancer year by year. The main clinical treatment for colorectal cancer is surgical resection, but surgery is traumatic, which results in a risk of postoperative complications [16, 17] and compromises the prognosis [18]. Predictive nursing is a new type of nursing method, which mainly refers to the comprehensive analysis of the patient's condition, the identification of potential risks in advance, and the application of effective nursing measures to prevent nursing risks and improve nursing efficiency [19]. In predictive nursing, psychological interventions and health education were provided to lessen the patients' pressure and eliminate their negative emotions for better treatment efficiency. The results of the present study showed that predictive nursing was associated with shorter operation time and hospital stay and less intraoperative blood loss versus conventional nursing, and patients given predictive nursing had a lower incidence of complications versus conventional nursing. There are different degrees of malnutrition in all patients before surgery, which affects the patient's physical condition. Individual dietary interventions are given in advance to increase the tolerance of the surgery and ensure a smooth surgery. Moreover, to achieve better surgical and nursing efficiency, the proficiency of nurses is critical, which serves to improve the patient's surgical condition, ameliorate the prognosis, reduce the incidence of adverse reactions, and accelerate the postoperative recovery. The results of the present study showed patients receiving predictive nursing were less anxious than those given conventional nursing. Moreover, the quality-of-life scores of the study group were elevated, and the social function, emotional function, cognitive function, role function, and physical function scores of the study group were all higher than those of the conventional group, which can be attributed to the fact that predictive nursing requires monitoring of patients' emotional changes and timely psychological interventions to reduce tension and fear, which can effectively prevent the muscle tension and metabolic disorders caused by negative emotions. All these were consistent with the results of previous research [20]. Furthermore, predictive nursing herein resulted in a higher nursing satisfaction versus conventional nursing, indicating that predictive nursing was well recognized by the patients. The reason may be that the nursing enhanced patients' knowledge of self-care and disease control, which contributes to improving their quality of life, so the patients were more satisfied with the nursing model.

Studies have shown that the use of traditional Chinese medicine (TCM) with chemotherapy or radiotherapy after colorectal cancer surgery can reduce the toxic side effects of radiotherapy, enhance immune function and improve the quality of life. On the basis of evidence-based treatment, TCM treatment adopts the principle of supporting righteousness and eliminating evil and achieves the effects of antirelapse and metastasis, thereby prolonging the survival and improving the survival quality. Therefore, TCM treatment is considered an important treatment method for postoperative patients with colorectal cancer. The innovative application of anticipatory care has good clinical guiding significance, but the limitation of this study is that a long-term follow-up investigation was absent to explore the disease-free survival time for patients, which will be conducted in future studies to obtain more clinical data.

## 5. Conclusion

Early predictive nursing for patients receiving colorectal cancer surgery can lower the incidence of complications, effectively improve the quality of life of patients, shorten the hospital stay, reduce the amount of bleeding, and enhance the satisfaction of patients.

## Figures and Tables

**Figure 1:** Comparison of nursing satisfaction of two groups of patients.

**Table 1:** Baseline data ($\bar{x}\pm s$).

Groups	n	Gender		Age		Course of disease	
		Male	Female	Range	Mean	Range	Mean
Routine group	65	37	28	42–73	57.45 ± 3.28	1–4	2.23 ± 0.28
Study group	65	36	29	41–75	57.68 ± 4.02	1–4	2.17 ± 0.56
*t*	—	—	—	—	0.357	—	0.773
*P* value	—	—	—	—	0.722	—	0.441

**Table 2:** Comparison of operation time, blood loss, and hospital stay between the two groups ($\bar{x}\pm s$).

Groups	n	Operation time (h)	Blood loss (ml)	Hospital stay (d)
Routine group	65	3.02 ± 0.78	81.51 ± 17.74	11.20 ± 2.14
Study group	65	2.35 ± 0.41	70.52 ± 16.52	9.32 ± 1.86
*t*	—	6.130	3.655	5.346
*P*	—	<0.001	<0.001	<0.001

**Table 3:** Comparison of complications between the two groups (%).

Groups	n	Bloating	Hypothermia	Wound infection	Subcutaneous emphysema	Lower extremity venous thrombosis	Total
Routine group	65	5 (7.69)	5 (7.69)	4 (6.15)	6 (9.23)	3 (4.62)	23 (35.38)
Study group	65	3 (4.62)	1 (1.54)	1 (1.54)	2 (3.08)	0 (0.00)	7 (10.76)
x^2^	—	11.093					
*P* value	—	0.001					

**Table 4:** Comparison of operation time, blood loss, and hospital stay between the two groups ($\bar{x}\pm s$).

		Routine group (*n* = 65)	Study group (*n* = 65)	t	*P* value
Social function	Before	64.48 ± 11.15	64.15 ± 11.74	0.164	0.870
	After	73.85 ± 13.54	83.51 ± 12.56	4.217	<0.001

Emotional function	Before	63.45 ± 10.55	63.51 ± 11.17	0.031	0.975
	After	72.54 ± 12.74	82.45 ± 9.15	5.094	<0.001

Cognitive function	Before	63.45 ± 11.17	63.78 ± 11.48	0.166	0.868
	After	72.48 ± 10.45	82.48 ± 10.46	5.453	<0.001

Role function	Before	63.78 ± 10.95	63.98 ± 10.65	0.106	0.916
	After	73.99 ± 14.51	84.43 ± 13.48	4.250	<0.001

Body function	Before	62.87 ± 10.91	62.12 ± 11.94	0.374	0.709
	After	72.45 ± 11.69	82.73 ± 9.67	5.463	<0.001

^*∗*^There is a difference between the two groups (*P* < 0.05).

## Data Availability

All the data generated or analyzed during this study are included in this published article.
